# Artificial Intelligence and Internet-of-Things Technology Application on Ideological and Political Classroom Teaching Reform

This article has been retracted.

**DOI:** 10.1155/2022/3496676

**Published:** 2022-06-30

**Authors:** Chang Cao

**Affiliations:** Henan Economy and Trade Vocational College, Zhengzhou, Henan 450046, China

## Abstract

We look at the current state of ideological and political classroom teaching based on artificial intelligence and the Internet of Things. We also look at the problems with traditional ideological and political classroom teaching in order to improve the effectiveness of classroom reform. Also, this paper reforms teaching based on the real world and builds a modern, intelligent system for teaching political and ideological ideas in the classroom. The ideological and political education system is built on the Internet of Things. It has three layers: the perception layer, the network layer, and the application layer. The system collects efficient ideological and political teaching activity data in real time through the Internet of Things and wireless networks, sends the data to the data center through the Internet, and then uses the collected data as the original data for applications, data mining, and modeling simulation. Lastly, this paper proves through simulation experiments and teaching experiments that the system built in this paper can be used to reform ideological and political education.

## 1. Introduction

At the moment, there are two kinds of intelligent teaching status analysis technology, depending on whether or not wearable devices are needed. One of them is based on wearable devices like EEG, eye trackers, and skin testers that measure how students' bodies are responding. Moreover, it judges the current student's classroom behavior state according to the frequency range of brain waves, eye movement, gaze direction, and changes in skin resistance [1]. Wearable technology is obtrusive and will unavoidably have an effect on the subjects. Therefore, there is a discrepancy between the obtained data and the actual classroom behavior of students. In addition, wearable technology is costly, cumbersome, and difficult to utilize, which makes it challenging to implement in actual classroom settings. The other is to collect video, image, voice, and other digital signals through cameras, microphones, and other equipment, and then extract information from these digital signals, such as student expressions, natural language, and body posture, and finally process, analyze, and merge the information to obtain the student's classroom behavior state [2]. The video image-based classroom student status analysis technology only needs to use the classroom camera system, so its cost is low, less intrusive, and has almost no impact on the student's learning process. Moreover, it can obtain student status information in real time, comprehensively and multi-dimensionally, so it has received extensive attention from major domestic and foreign technology companies and research institutions [3].

However, when the current student state analysis technology based on video images is applied to a real classroom environment, there are still some problems to be broken through. First of all, the current video analysis technology is mainly oriented to “less but precise” application scenarios. However, due to the limitation of teaching hardware resources, the real nature classroom has a large number of learners and a limited number of cameras. How to quickly and accurately analyze the learning status of students in a complex environment with multiple scales, multiple angles, and multiple illuminations? This paper investigates the use of artificial intelligence (AI) and the Internet of Things (IoT) technology in ideological and political classroom teaching, and it also constructs an intelligent teaching system that is based on actual teaching conditions in order to improve the efficiency of ideological and political classroom teaching.

## 2. Related Work

In recent years, the widespread use of new-generation information technologies, such as mobile Internet, the Internet of Things, cloud computing, big data, and artificial intelligence, has had a dramatic effect on all facets of social life. “There will be no modernization in the absence of informatization.” The consensus in the education community is that “information technology has a revolutionary effect on the evolution of education.” Under the guidance and promotion of a series of educational informatization policies in my country, numerous schools are actively creating conditions to upgrade the construction and application of educational informatization, and are beginning to explore feasible means to realize smart education, such as constructing smart classrooms and smart campuses.

For the smart learning environment, literature [4] believes that from the perspective of the designer, it is the technical support of smart education. As a new type of learning environment, it needs to be guided by many advanced ideas and theories of learning, teaching, management, and utilization, and supported by appropriate modern information technology, learning tools, learning resources, and learning activities. At the same time, it needs to fully perceive the learning situation information to obtain new data or conduct scientific analysis and data mining on the historical data formed by the learners in the learning process. After identifying learners' characteristics and learning situations, the system must generate optimally adapted learning tasks and activities, guide and assist learners in making correct decisions, and effectively promote the development of intelligent capability and the emergence of intelligent actions.

The literature [5] put forward the viewpoints of the transformation from the digital learning environment to the smart learning environment, and the smart learning environment is the high-end form of the ordinary digital learning environment. On the basis of analyzing and synthesizing other scholars' ideas of smart learning environment, the concept of “smart learning environment” was put forward. In other words, it is a learning environment or activity space that can perceive learning situations, identify learner characteristics, provide appropriate learning resources and convenient interactive tools, automatically record learning processes, and evaluate learning outcomes in order to promote effective learning among learners. The literature [6] further clarified the relationship between the technical support and the components of the smart learning environment, that is, the smart learning environment has four components (learning resources, smart tools, learning communities, and teaching communities) and four technical characteristics (record the process, identify the situation, perceive the environment, and connect with the community). Its purpose is to promote easy, engaged, and effective learning for learners. The composition of the smart learning environment should be related to specific teaching methods and learning methods, and there is no unified and general smart learning environment.

The literature [7] deconstructed smart education from the perspective of system, technology, and function realization, and conducted research on the technology integration in the smart education system and the technology drive of smart features. Moreover, it believed that smart education is a complex ecosystem composed of multiple educational activities, processes, and functional technical modules and mutual feedback, that is, smart education system and functional model. The model is mainly composed of four parts: smart learning with learners as the main body, smart teaching with teachers as the main body, smart education resources and technical environment (smart education cloud) from the perspective of developers, and smart education system from the perspective of managers. The literature [8] pointed out the key technologies of smart education, described the features and application scenarios of smart education brought by technology, and gave suggestions for the integration and development of smart education technologies. On the basis of studying the development strategy and path selection of smart education in my country, the connotation and characteristics of smart education, literature [9] proposed a design plan for the system architecture and key supporting technologies of smart education from the perspective of system engineering and technology realization. Moreover, it systematically discussed the construction of a smart education environment (a smart campus that supports school education and a learning smart city that supports life-long education), the construction of smart learning content library (including learning resource library, open curriculum library, and management information library), and the comprehensive application of smart technologies (including cloud computing, big data, ubiquitous networks, and augmented reality), and how to provide smart services for teachers, students, parents, education administrators, etc. (including smart teaching, smart learning, smart communication, smart management, and smart evaluation). Simultaneously, it was believed that smart education necessitates strong information technology application capabilities in teachers and students, and that the rational, effective, and innovative application of information technology can promote the entire design, implementation, and evaluation of teaching and learning activities before, during, and after class.

Literature [10] uses “understanding the basic schema of smart education” to reveal the internal relationship between smart education, smart environment, and smart teaching methods, and proposes that smart education should be supported by smart learning environment (designer's perspective). Using smart teaching methods as a catalyst (teacher's perspective), with smart learning as the fundamental cornerstone (learner's perspective), smart education in an information environment refers to education that develops students' smart abilities under the support of information technology, and aims to use appropriate Information technology to build a smart learning environment (technical innovation), use smart teaching methods (method innovation), and promote learners to carry out smart learning (practical innovation), so as to cultivate a good value orientation, higher thinking quality, and strong performance. Competent intelligent talents (to change the concept of talents, we must cultivate intelligent talents who are good at learning, good at collaboration, good at communication, good at research and judgment, good at creativity, and good at solving complex problems), implement the concept of wisdom education (idea innovation), and deepen and improve information Quality education in the age, knowledge age, and digital age. According to the literature [11], the basic connotation of wisdom education in the information age is by constructing a smart learning environment and using smart teaching methods to promote learners' smart learning, thereby enhancing their expectations of success, that is, cultivating people with high intelligence and creativity and using Appropriate technology intelligently participates in various practical activities and continuously creates products and values, so as to realize the smart and smart adaptation, shaping and selection of the learning environment, living environment, and working environment.

## 3. IoT Node Algorithm

Sampling- and filtering-based signal strength resolution (SF-SSR) adopts the sampling and filtering ideas in MCL and combines the ideas of synthesis and decomposition of physical forces. It is based on RSS ranging technology and belongs to a distance-based positioning algorithm [12].

The main physical ideas are:

1. The force between objects is interacting, and the force is a vector with two magnitude and direction elements.
2. In WSN, the process of a beacon node transmitting and receiving an RSS signal, and a mobile node receiving and transmitting an RSS signal while moving, is regarded as the interaction of force between the objects.
3. The signal vector between the mobile node and the beacon node, which includes the two elements of the signal strength value and the receiving angle between the two.
4. Force decomposition refers to the process of determining the component force of a known force. 2nd Definition (vector decomposition angle). The process of decomposing the signal vector between the mobile node and the beacon node on the *X* and *Y* axes is known as signal vector decomposition, and the decomposed angle is known as vector decomposition angle.

**Definition 1 .**

(signal sum vector). The signal sum vector is the signal vector obtained by decomposing and synthesizing the signal vector between the mobile node and the beacon node on the *X* and *Y* axes.

The SF-SSR algorithm uses RSS ranging technology to calculate the distance between the mobile node and the signal strength between the beacon node within the communication radius of one hop. Select 2 beacon nodes with the strongest signal strength to establish a rectangular coordinate system with the mobile node, and then use 3 beacon nodes with the strongest signal strength to perform initial positioning of the mobile node, using the initial positioning position as the center of the circle and the center of the network. The maximum and minimum positioning error is the circle formed by the radius as the sampling area. The combined vector of the mobile node and the sample point relative to the two beacon nodes with larger signal strength is calculated, respectively, and finally the sample points are screened according to the specified filter conditions to realize the movement in the positioning of the node [13].

Figure 1 is a system framework diagram of the SF-SSR algorithm.

The communication chip of the existing sensor node (such as Chipcon's CC2431) has the function of wireless communication, and can complete the RSS measurement while receiving data, and does not need to configure additional hardware, which meets the low-power and low-cost requirements of WSN.

We assume that the one-hop communication range of all nodes in the network is *r*, which corresponds to the range of direct communication, that is, the communication radius is *r*. The beacon nodes within the one-hop communication range of the mobile node *L*_1_ at time *t* are screened, and they are sorted according to the magnitude of the received signal strength to form a beacon node sequence {*S*_*i*_^*t*^}, *i*=1,2,3,…, *k* (*k* represents the number of beacon nodes within the one-hop communication range). According to formula (1), it can be seen that the distance between the beacon node and the mobile node is inversely proportional to the signal strength. In other words, the shorter the distance between the beacon node and the mobile node, the more consistent the network environment and natural environment, where the beacon node and mobile node are located. The impact of external conditions on signal strength and network range error is comparable. Therefore, the algorithm selects *S*_1_^*t*^ and *S*_2_^*t*^ in the beacon node sequence {*S*_*i*_^*t*^} whose signal strength values are at the top, and takes *S*_1_^*t*^ as the origin and the connection of *S*_1_^*t*^ and *S*_2_^*t*^ as the *x* axis to establish a rectangular coordinate system. After selecting *S*_1_^*t*^, *S*_2_^*t*^, *S*_3_^*t*^ in the beacon node sequence {*S*_*i*_^*t*^}, according to the empirical formula [14]:

(1) $$\begin{array}{c} P_{r}\left(d\right)=P_{0}\left(d_{0}\right)+10n_{p}\mathrm{lg}\left(\frac{d}{d_{0}}\right)+X_{0}. \end{array}$$

In the formula, *P*_*r*_(*d*) represents the signal strength of the wireless signal after the distance *d*, *P*_0_(*d*_0_) represents the reference signal strength at the reference distance *d*_0_, and *d* represents the distance between the transmitting end and the receiving end, *n*_*p*_ represents the path loss index, *X*_0_ represents the random noise with a mean value of 0 and following a Gaussian distribution.

It can be deduced from equation (1) that if the signal strength value *p*_1*i*_^*t*^ between *S*_1_^*t*^ and *L*_1_ is given, the maximum likelihood of the ranging distance *d*_1*i*_^*t*^ between *n* and *b* is estimated as [15]:

(2) $$\begin{array}{c} d_{1i}^{t}=d_{0}{\left(\frac{p_{1i}^{t}}{P_{0}\left(d_{0}\right)}\right)}^{\left(1/n_{p}\right)}. \end{array}$$

In the same way, from the signal strength value *p*_2*i*_^*t*^, *p*_3*i*_^*t*^ between *S*_2_^*t*^, *S*_3_^*t*^ and *L*_*i*_, the distance *d*_2*i*_^*t*^, *d*_3*i*_^*t*^ between *S*_2_^*t*^, *S*_3_^*t*^ and *L*_*i*_ can be calculated.

According to the distance measurement between *S*_1_^*t*^, *S*_2_^*t*^, *S*_3_^*t*^ and *L*_*i*_, the approximate position $L_{i}^{t}\left({\hat{x}}^{t},{\hat{y}}^{t}\right)$ of the node can be determined using the trilateral positioning method, and thus the quadrant of *L*_*i*_ can be judged.

As shown in Figure 2, the angle between the signal vector $\bar{S_{1}^{t}L_{i}^{t}},\bar{S_{2}^{t}L_{i}^{t}}$ and the *x*-axis is ∠*α*, ∠*β*. The vector decomposition angle is based on the origin, that is, the beacon node *S*_1_^*t*^, and it is specified that the counterclockwise rotation on the top of the *x*-axis is 0° to 180°, and the counterclockwise rotation on the bottom of the *x*-axis is −180° to 0°. We explain the vector decomposition angle of the signal vector $\bar{S_{1}^{t}L_{i}^{t}},\bar{S_{2}^{t}L_{i}^{t}}$ in two cases. Case 1: when ∠*α*, ∠*β* ∈ [0°, 180°], as shown in Figure 2 (a), the decomposition angle of the signal vector $\bar{S_{1}^{t}L_{i}^{t}}$ is ∠*α*, and the decomposition angle of the signal vector $\bar{S_{2}^{t}L_{i}^{t}}$ is ∠*β*. Case 2: when ∠*α*, ∠*β* ∈ [−180°, 0°], as shown in Figure 2 (b), the decomposition angle of the signal vector $\bar{S_{1}^{t}L_{i}^{t}}$ is ∠*α*, and the decomposition angle of the signal vector $\bar{S_{2}^{t}L_{i}^{t}}$ is −*π* − ∠*β* [16].

We set the coordinates of *S*_1_^*t*^, *S*_2_^*t*^ as (*x*_1_, *y*_1_), (*x*_2_, *y*_2_) respectively, and use the distance formula between two points to find the distance *d*_12_ between *S*_1_^*t*^, *S*_2_^*t*^.

(3) $$\begin{array}{c} d_{12}=\sqrt{{\left(x_{1}-y_{1}\right)}^{2}{\left(x_{2}-y_{2}\right)}^{2}}. \end{array}$$

In Δ*S*_1_^*t*^*L*_*i*_^*t*^*S*_2_^*t*^, we use the law of cosines and the induced formula to find:

(4) $$\begin{array}{c} \cos\;\alpha =\frac{{\left(d_{1i}^{t}\right)}^{2}+{\left(d_{12}\right)}^{2}+{\left(d_{2i}^{t}\right)}^{2}}{2d_{1i}^{t}d_{12}}, \end{array}$$

(5) $$\begin{array}{c} \sin\;\alpha ={\left(-1\right)}^{h}\sqrt{1-\;\cos^{2}\;\alpha ,h=1,2}. \end{array}$$

In the same way, cos  *β*, sin  *β* is found.

According to the vector decomposition angle of *L*_*i*_ and *S*_1_^*t*^, *S*_2_^*t*^, the signal resultant vector of the mobile node on the *x* and *y* axis is calculated.

(6) $$\begin{array}{c} {\bar{x}}^{t}=\bar{S_{1}^{t}L_{i}^{t}}\cos\;\alpha +\bar{S_{2}^{t}L_{i}^{t}}\cos\left({\left(-1\right)}^{h}\pi -\beta \right),\\ {\bar{y}}^{t}=\bar{S_{1}^{t}L_{i}^{t}}\sin\;\alpha +\bar{S_{2}^{t}L_{i}^{t}}\sin\left({\left(-1\right)}^{h}\pi -\beta \right),\\ h=1,2. \end{array}$$

In case 1, the value of *h* in equations (5) and (6) is 2. In case 2, the value of *h* in formulas (5) and (6) is 1.

In the real world, signal propagation is easily influenced by reflection, scattering, and diffraction, so the distance accuracy of the RSS range technology is not particularly great. Inaccurate node positioning and positioning mistakes will result from using the m-edge positioning method. The positioning error is the difference between the actual and projected positions. If the error range can be calculated, then the genuine position can also be determined. The SF-SSR technique employs the network's highest and minimum positional errors to determine the ring sampling area [17].

Since the mobile node and the beacon node {*S*_*i*_^*t*^} are in the same network environment, their RSS ranging technology positioning error is the same. Then, the beacon node sequence {*S*_*i*_^*t*^} can be used to calculate the maximum and minimum positioning errors in the network to determine the area where *L*_*i*_ is located. The beacon node in {*S*_*i*_^*t*^} calculates its own coordinate $\left\{\left(\hat{x},\hat{y}\right)\right\},i=1,2,3,\ldots ,k$ through the coordinates of its neighbor beacon nodes and the RSS ranging information, and then uses equation (7) to obtain the positioning error *e*_*i*_ according to its actual position.

(7) $$\begin{array}{c} e_{i}=\frac{\sqrt{{\left(\hat{x}-x_{i}\right)}^{2}+{\left(\hat{y}-y_{i}\right)}^{2}}}{r},\;i=1,2,3,\ldots ,k. \end{array}$$

If the maximum positioning error is set to *e*_max_, then:

(8) $$\begin{array}{c} e_{\max}=\max\left(e_{i}\right),\;i=1,2,3,\ldots ,k. \end{array}$$

If the minimum positioning error is *e*_min_, then:

(9) $$\begin{array}{c} e_{\min}=\min\left(e_{i}\right),\;i=1,2,3,\ldots ,k. \end{array}$$

We set up the sampling area with the position *L*_*i*_^*t*^ of the time *t* obtained by the trilateral positioning as the center of the circle and with *re*_max_ and *re*_min_ as the radius, as shown in Figure 3. In the figure, the gray filled area is the sampling area of the SF-SSR algorithm.

V sample points $\tilde{s^{t}}\left(\tilde{x_{j}},\tilde{y_{j}}\right),j=1,2,\ldots ,v$ are randomly distributed. Since the sample point is a virtual point, it can be inversely calculated from the distance between $\tilde{s^{t}}$ and *S*_1_^*t*^, *S*_2_^*t*^ using equation (2) to obtain the signal strength of the sample point, and then resolve the different situations of the angle according to the signal vector [18].

According to formulas (3) and (5), the signal resultant vector $\bar{{\tilde{x_{j}}}^{t}},\bar{{\tilde{y_{j}}}^{t}},j=1,2,\ldots ,v$ on the *x*-axis and *y*-axis of $\tilde{s^{t}}\left(\tilde{x_{j}},\tilde{y_{j}}\right),j=1,2,\ldots ,v$ relative to *S*_1_^*t*^, *S*_2_^*t*^ is calculated.

**Theorem 1 .**

The position of *L*_*i*_ at time *r* must be inside or on a circle with *L*_*i*_^*t*^ as the center and *re*_max_ and *re*_min_ as radii.

**Proof**

If the position of *L*_*i*_ at time *t* is set to (*x*^*t*^, *y*^*t*^), judging the relationship between a point and the circle can be transformed into judging the relationship between the distance from the point to the center of the circle and the radius of the circle. If the distance between the position (*x*^*t*^, *y*^*t*^) of *L*_*i*_ and the center of the circle at time *t* is $D=\sqrt{{\left({\hat{x}}^{t}-x^{t}\right)}^{2}+{\left({\hat{y}}^{t}-y^{t}\right)}^{2}}$, and the positioning error of *L*_*i*_ at this time is $e=\sqrt{{\left({\hat{x}}^{t}-x^{t}\right)}^{2}+{\left({\hat{y}}^{t}-y^{t}\right)}^{2}}/r$, then *D*=*er*. The minimum and maximum errors in the network have *e*_min_ ≤ *e* ≤ *e*_max_, so there is *re*_min_ ≤ *re* ≤ *re*_max_.

The SF-SSR algorithm mainly uses the filtering method with the smallest signal resultant vector difference to filter the sample points in the sampling area, and screen the sample points. First, the algorithm filters out the sample points $\tilde{s_{1}^{t}}\left(\tilde{x_{j}},\tilde{y_{j}}\right),j=1,2,\ldots ,m$ in the same direction as $\bar{{\tilde{x_{j}}}^{t}},\bar{{\tilde{y_{j}}}^{t}},j=1,2,\ldots ,m$ respectively, in $\bar{{\tilde{x_{j}}}^{t}},\bar{{\tilde{y_{j}}}^{t}},j=1,2,\ldots ,v$ (m represents the number of sample points selected according to the direction). Secondly, the algorithm compares the size of $\bar{{\tilde{x_{j}}}^{t}},\bar{{\tilde{y_{j}}}^{t}},j=1,2,\ldots ,m$ modulus with ${\bar{x}}^{t}$, ${\bar{y}}^{t}$ modulus.

(10) $$\begin{array}{c} {\hat{\varphi }}_{j}^{x}=\sqrt{{\left(\left|{\bar{x}}^{t}\right|-\left|{\bar{\tilde{x}}}_{j}^{t}\right|\right)}^{2}},\\ {\hat{\varphi }}_{j}^{y}=\sqrt{{\left(\left|{\bar{y}}^{t}\right|-\left|{\bar{\tilde{y}}}_{j}^{t}\right|\right)}^{2}},\\ j=1,2,\ldots ,m. \end{array}$$

Since ${\bar{x}}^{t},{\bar{y}}^{t}$ , $\bar{{\tilde{x_{j}}}^{t}},\bar{{\tilde{y_{j}}}^{t}},j=1,2,\ldots ,v$ is unique at time *t*, the coordinates of *L*_*i*_ and *s*_1_^*t*^ correspond to ${\bar{x}}^{t},{\bar{y}}^{t}$ and $\bar{{\tilde{x_{j}}}^{t}},\bar{{\tilde{y_{j}}}^{t}},j=1,2,\ldots ,v$ one-to-one:

(11) $$\begin{array}{c} {\hat{\varphi }}_{\min}^{x}=\min\left({\hat{\varphi }}_{j}^{x}\right),\\ {\hat{\varphi }}_{\min}^{y}=\min\left({\hat{\varphi }}_{j}^{y}\right),\\ j=1,2,\ldots ,m. \end{array}$$

We set the coordinate set of $\tilde{s_{1}^{t}}$ corresponding to ${\hat{\varphi }}_{\min}^{x},{\hat{\varphi }}_{\min}^{y}$ as $\left(\tilde{x_{j}},\tilde{y_{j}}\right),j=1,2,\ldots ,w$ (w represents the number of sample points filtered by the minimum value), and the coordinate of *L*_*i*_ at time *t* is $\left(\tilde{x_{j}},\tilde{y_{j}}\right)$. After many experiments, it is found that when the mean value of the coordinate set of $\tilde{s_{1}^{t}}$ is the mobile node coordinate, the positioning error is the smallest. Then, there is [19]:

(12) $$\begin{array}{c} {\tilde{x}}^{t}=\frac{1}{w}\sum_{j}^{n}\tilde{x_{i}},\\ {\tilde{y}}^{t}=\frac{1}{w}\sum_{j}^{n}\tilde{y_{i}},\\ j=1,2,\ldots ,w. \end{array}$$

**Theorem 2 .**

At time *t*, ${\bar{x}}^{t},{\bar{y}}^{t}$ , $\bar{{\tilde{x}}^{t}},\bar{{\tilde{y}}^{t}},j=1,2,\ldots ,v$ is unique.

**Proof**

We take *L*_*i*_ as an example. At time *t*, the coordinate of the component vector obtained by decomposing the signal vector $\overset{⟶}{s_{j}^{t}L_{i}^{t}}\left(j=1,2\right)$ along the *x*-axis is denoted as $\left({\bar{x}}^{'t},0\right),\left({\bar{x}}^{'\prime t},0\right)$, the coordinate of the signal component along the *y*-axis direction is denoted as $\left({\bar{y}}^{'t},0\right),\left({\bar{y}}^{'\prime t},0\right)$, and the resultant vector coordinate of the *x*-axis and *y*-axis of *b* is denoted as $\left({\bar{x}}^{'t}+{\bar{x}}^{'\prime t},0\right),\left(0,{\bar{y}}^{'t}+{\bar{y}}^{'\prime t}\right)$. Since there is a one-to-one correspondence between the vector and its coordinate representation, the uniqueness of $\left({\bar{x}}^{'t}+{\bar{x}}^{'\prime t},0\right),\left(0,{\bar{y}}^{'t}+{\bar{y}}^{'\prime t}\right)$ is proved. There are two cases. Case 1: ${\bar{x}}^{'t},{\bar{x}}^{'\prime t}$ has an opposite sign, that is, when *S*_1_^*t*^, *S*_2_^*t*^ is on the opposite side of *L*_*i*_, as shown in Figure 4, the value of $\left|{\bar{x}}^{'t}\right|+\left|{\bar{x}}^{'\prime t}\right|$ is unique. That is, regardless of the mapping coordinates of the component vector of the signal vector $\bar{S_{j}^{t}L_{i}^{t}}\left(j=1,2\right)$ in the *x*-axis direction, as long as *S*_1_^*t*^, *S*_2_^*t*^ is determined, the sum of its absolute values is always fixed. The question is transformed into whether there is a unique set of ${\bar{x}}^{'t},{\bar{x}}^{'\prime t}$ whose sum is *C*_1_ and difference is *C*_2_ under the premise that $\left|{\bar{x}}^{'t}\right|+\left|{\bar{x}}^{'\prime t}\right|$ is fixed, that is, it proves whether the inhomogeneous linear equation system [20].

(13) $$\begin{array}{c} \left\{\begin{array}{c} {\bar{x}}^{'t}+{\bar{x}}^{'\prime t}=C_{1},\\ {\bar{x}}^{'t}-{\bar{x}}^{'\prime t}=C_{2}, \end{array}\right. \end{array}$$

has a unique solution. The coefficient matrix of this linear equation system is

(14) $$\begin{array}{c} A=\left(\begin{array}{cc} 1 & 1\\ 1 & -1 \end{array}\right). \end{array}$$

Its augmented matrix is

(15) $$\begin{array}{c} \bar{A}=\left(\begin{array}{cc} 1 & 1C_{1}\\ 1 & -1C_{2} \end{array}\right),\\ r\left(A\right)=r\left(\bar{A}\right)=2. \end{array}$$

Therefore, the system of equations has a solution and a unique solution. Case 2: ${\bar{x}}^{'t},{\bar{x}}^{'\prime t}$ is the same sign, that is, when the beacon node *S*_1_^*t*^, *S*_2_^*t*^ is on the same side of the mobile node *L*_*i*_, as shown in Figure 4, ${\bar{x}}^{'t},{\bar{x}}^{'\prime t}$ is both positive or negative, and ${\bar{x}}^{'t}-{\bar{x}}^{'\prime t}$ is unique. That is, no matter how much the component vector of $\bar{S_{1}^{t}L_{i}^{t}},\bar{S_{2}^{t}L_{i}^{t}}$ is in the *x*-axis direction, as long as *S*_1_^*t*^, *S*_2_^*t*^ is determined, ${\bar{x}}^{'t}-{\bar{x}}^{'\prime t}$ is a fixed value. Under this condition, the problem is also transformed to prove that formula (13) has a unique solution, ibid. As shown in Figure 4, if $\left(0,{\bar{y}}^{\prime t}\right),\left(0,{\bar{y}}^{\prime \prime t}\right)$ is both positive or negative, the value of $\left(0,{\bar{y}}^{\prime t}+{\bar{y}}^{\prime \prime t}\right)$ is also unique, that is, ${\bar{x}}^{t},{\bar{y}}^{t}$ is unique. That is to say, as long as the position of *L*_*i*_ is determined, the signal resultant vector of *S*_1_^*t*^, *S*_2_^*t*^ relative to *L*_*i*_ is unique. Similarly, as long as the position of $\bar{S_{j}^{t}}$ is determined, the signal resultant vector of the sample point relative to *S*_1_^*t*^, *S*_2_^*t*^ is unique [21].

## 4. Ideological and Political Classroom Teaching System based on Artificial Intelligence and Internet of Things Technology

This article combines the actual needs of ideological and political classroom teaching, analyzes the existing problems in traditional ideological and political classroom teaching, reforms the teaching in accordance with the actual situation, and builds a modern intelligent ideological and political classroom teaching system. The perception layer, the network layer, and the application layer are all components of the structure of the ideological and political education system that is represented by the Internet of Things. Based on the overall requirements of the IoT teaching development platform, this paper proposes a more optimized overall system architecture, as shown in Figure 5 [22].

The cloud architecture design of the ideological and political teaching development system based on the Internet of Things is shown in Figure 6.

The overall structure of the teaching platform is shown in Figure 7. The platform collects real-time data of school ideological and political teaching activities through the Internet of Things and wireless networks, then transmits the data to the data centers through the Internet, and finally uses the collected data as the original data for application, data mining, and modeling simulation based on the data that was collected through the platform. The Internet of Things layer and the data center layer are connected by the wireless network and the campus network. These networks not only play the role of data storage and data transfer, but they also provide network services for the operation of platforms and the collection of data. It serves as the primary nerve center of the entire platform [23].

## 5. Performance Verification of Ideological and Political Classroom Teaching System based on Artificial Intelligence and Internet of Things Technology

The purpose of this article is to develop an intellectual and political education platform by utilizing technologies such as the Internet of Things and artificial intelligence. Using the technology that is available through the Internet of Things, the system is able to swiftly improve the acquisition and transmission of educational resources. This article primarily investigates the transmission efficiency of ideological and political teaching resources in the Internet of Things node, as well as the evaluation of the effects of ideological and political teaching, in order to execute the system performance verification.

This article combines simulation experiments to construct the Internet of Things nodes in this system. It then collects ideological and political teaching resources through the network, transmits teaching resources through a model of the Internet of Things node, and calculates the transmission efficiency of those teaching resources, as shown in Table 1 and Figure 8.

From the above research results, we can see that the ideological and political classroom teaching system based on artificial intelligence and Internet of Things technology constructed in this paper has a good teaching resource transmission effect. After that, this paper evaluates its teaching effect through experimental teaching methods, and counts the evaluation results, as shown in Table 2 and Figure 9.

Through the above analysis, it can be seen that the ideological and political teaching system based on artificial intelligence and Internet of Things technology constructed in this paper has good teaching effects and can effectively promote the reform of ideological and political classroom teaching.

## 6. Conclusion

Through the use of modeling and simulation software, this study creates a simulation model, then uses that model to perform research and analysis on the data acquired regarding the ideological and political teaching activities that take place in colleges and universities. In addition, this article makes use of intuitive and visual means to reflect the actual situation of ideological and political teaching activities that take place in colleges and universities. As a result, instructors will have a much easier time comprehending the current state of the physical education system. In addition, this paper provides an overview of the ideological and political education provided in colleges and universities by analyzing the situation depicted by the simulation model, identifying the issues that currently exist, and outlining potential solutions in order to enhance the quality of ideological and political education provided in academic institutions.

The design of the educational platform not only takes into account the fundamental circumstances of ideological and political instruction in academic institutions of higher learning, but it also takes into account the implementation of cutting-edge information technology. This is done so in order to maximize the efficiency in the classroom. At the same time, it not only ensures that the platform has complete functions and advanced technology, but also that it is an innovation and breakthrough to the traditional teaching platform, which is conducive to better assisting the ideological and political teaching of colleges and universities. In addition, it ensures that the platform has complete functions and advanced technology. It is conducive to improving the relationship between teachers and students, strengthening the guidance of the ideological and political learning process in universities, and playing an important role in improving student learning efficiency and teaching quality. In addition, this is not only an improvement to the original teaching platform, but it is also real-time collection of ideological and political teaching activity data in colleges and universities.

## Figures and Tables

**Figure 1:** SF-SSR system framework diagram.

**Figure 2:** Vector decomposition angle of mobile node.

**Figure 3:** Sampling area of SF-SSR.

**Figure 4:** The beacon node is on the opposite side or the same side of the mobile node.

**Figure 5:** The overall architecture of the ideological and political teaching development system based on the Internet of Things.

**Figure 6:** Cloud architecture design.

**Figure 7:** The overall architecture of an ideological and political teaching platform based on the Internet of Things.

**Figure 8:** Statistics diagram of the resource transmission effect of IoT nodes.

**Figure 9:** Statistical diagram of the evaluation of the teaching effect of the ideological and political teaching system based on artificial intelligence and Internet of things technology.

**Table 1:** Statistics table of the resource transmission effect of IoT nodes.

Num	Resource transfer	Num	Resource transfer	Num	Resource transfer
1	95.80	30	97.22	59	92.93
2	91.51	31	91.10	60	91.09
3	93.93	32	92.37	61	94.73
4	92.31	33	89.80	62	96.93
5	92.38	34	95.15	63	95.80
6	96.48	35	95.54	64	93.46
7	92.74	36	92.30	65	96.59
8	89.20	37	97.71	66	97.70
9	93.38	38	95.85	67	92.96
10	95.76	39	97.35	68	92.97
11	96.42	40	97.99	69	96.99
12	90.14	41	97.00	70	92.00
13	94.10	42	94.91	71	91.11
14	93.03	43	89.93	72	93.17
15	92.03	44	96.02	73	96.15
16	92.60	45	95.09	74	89.68
17	97.00	46	94.74	75	95.76
18	94.50	47	96.58	76	96.02
19	89.64	48	92.69	77	90.42
20	96.42	49	94.42	78	93.29
21	93.85	50	95.18	79	97.91
22	96.51	51	90.03	80	89.33
23	97.03	52	92.30	81	90.22
24	97.58	53	97.95	82	96.33
25	96.71	54	95.74	83	93.06
26	92.65	55	97.39	84	94.26
27	90.73	56	92.89	85	92.31
28	91.00	57	90.87	86	91.84
29	97.01	58	90.41		

**Table 2:** Statistical table of the evaluation of the teaching effect of the ideological and political teaching system based on artificial intelligence and Internet of things technology.

Num	Teaching evaluation	Num	Teaching evaluation	Num	Teaching evaluation
1	93.17	30	91.43	59	84.88
2	92.28	31	90.35	60	88.85
3	90.69	32	89.33	61	81.68
4	83.67	33	84.19	62	86.96
5	91.65	34	89.09	63	91.85
6	84.19	35	82.32	64	89.84
7	93.55	36	87.02	65	93.47
8	83.80	37	84.82	66	83.64
9	81.23	38	90.52	67	86.58
10	93.11	39	82.17	68	81.62
11	81.23	40	86.19	69	91.47
12	88.63	41	85.61	70	81.72
13	82.18	42	82.45	71	84.33
14	85.45	43	86.00	72	89.21
15	81.09	44	92.57	73	87.43
16	84.92	45	89.20	74	91.72
17	82.77	46	81.20	75	82.91
18	82.61	47	88.76	76	82.57
19	93.37	48	90.05	77	87.08
20	82.43	49	82.80	78	86.70
21	89.97	50	84.09	79	90.12
22	92.31	51	91.99	80	85.46
23	81.56	52	91.25	81	85.05
24	89.45	53	88.72	82	88.77
25	84.58	54	86.62	83	87.98
26	90.09	55	89.42	84	81.65
27	90.69	56	91.89	85	86.28
28	90.49	57	92.32	86	81.58
29	83.88	58	87.30		

## Data Availability

The data used to support the findings of this study are available from the author upon request.
